This article has been retracted.

# Detection of 3D Arterial Centerline Extraction in Spiral CT Coronary Angiography

**DOI:** 10.1155/2021/2670793

**Published:** 2021-08-21

**Authors:** Wenjuan Cai, Yanzhe Wang, Liya Gu, Xuefeng Ji, Qiusheng Shen, Xiaogang Ren

**Affiliations:** ^1^Changshu Hospital of Chinese Medicine, Changshu 215516, Jiangsu, China; ^2^School of Information and Control Engineering, China University of Mining and Technology, Xuzhou 221116, Jiangsu, China

## Abstract

This paper presents an in-depth study and analysis of the 3D arterial centerline in spiral CT coronary angiography, and constructs its detection and extraction technique. The first time, the distance transform is used to complete the boundary search of the original figure; the second time, the distance transform is used to calculate the value of the distance transform of all voxels, and according to the value of the distance transform, unnecessary voxels are deleted, to complete the initial contraction of the vascular region and reduce the computational consumption in the next process; then, the nonwitnessed voxels are used to construct the maximum inner joint sphere model and find the skeletal voxels that can reflect the shape of the original figure. Finally, the skeletal lines were optimized on these initially extracted skeletal voxels using a dichotomous-like principle to obtain the final coronary artery centerline. Through the evaluation of the experimental results, the algorithm can extract the coronary centerline more accurately. In this paper, the segmentation method is evaluated on the test set data by two kinds of indexes: one is the index of segmentation result evaluation, including dice coefficient, accuracy, specificity, and sensitivity; the other is the index of clinical diagnosis result evaluation, which is to refine the segmentation result for vessel diameter detection. The results obtained in this paper were compared with the physicians' labeling results. In terms of network performance, the Dice coefficient obtained in this paper was 0.89, the accuracy was 98.36%, the sensitivity was 93.36%, and the specificity was 98.76%, which reflected certain advantages in comparison with the advanced methods proposed by previous authors. In terms of clinical evaluation indexes, by performing skeleton line extraction and diameter calculation on the results obtained by the segmentation method proposed in this paper, the absolute error obtained after comparing with the diameter of the labeled image was 0.382 and the relative error was 0.112, which indicates that the segmentation method in this paper can recover the vessel contour more accurately. Then, the results of coronary artery centerline extraction with and without fine branch elimination were evaluated, which proved that the coronary artery centerline has higher accuracy after fine branch elimination. The algorithm is also used to extract the centerline of the complete coronary artery tree, and the results prove that the algorithm has better results for the centerline extraction of the complete coronary vascular tree.

## 1. Introduction

The growth of urban economies and the accelerated aging of the population, the prevalence of poor lifestyles, and the continued growth of risk factors that induce cardiovascular disease make it the number one cause of death in humans. According to World Health Organization statistics, in 2018, more than 17.5 million people died of heart-related diseases worldwide, accounting for 31% of the total death population. Among them, more than 7.4 million people suffered from coronary heart disease, which is 42% of all deaths from heart disease. Initial results have been achieved in the treatment of heart-related diseases, but the overall situation remains grim. In recent years, the total number of diseases and deaths from heart-related diseases has continued to increase in our country [1]. It is estimated that presently 290 million people are afflicted with heart-related diseases within our country, close to 21% of the total population. Among these patients, the vast majority suffer from hypertension, amounting to 270 million, and the population suffering from coronary heart disease amounts to 11 million [2]. Heart-related diseases account for 40% of the composition of the population's mortality factors, more than other diseases such as cancer. Experts predict that the population suffering from heart-related diseases will continue to increase in the next 10 years, and the burden of this disease is increasing. Therefore, how to effectively combat heart disease has become a serious issue. If an accurate diagnosis system can be established for heart diseases, targeted treatment can be implemented, and it will be of great importance to reduce the mortality rate due to heart diseases and thereby improve people's quality of life. With the advancement of technology in the field of medical image processing, its role in research and practice is becoming increasingly prominent [3]. Through the combination of computer science, mathematics, and imaging, medical images are analyzed to help locate lesions and improve the speed and accuracy of clinical diagnosis. In the analysis of coronary morphology, the extraction of the vascular tree is a fundamental problem. Accurate segmentation is a prerequisite for describing vascular geometric information and plays a key role in objectively and accurately assessing the extent of vascular lesions [4]. Most coronary vascular segmentation methods are for single-frame (static) images and are a well-established and effective method for helping to identify vascular lesions, but the accuracy of diagnostic results is compromised by temporal limitations that result in a lack of disease information. Therefore, describing the dynamic motion and changes of the vascular tree in the images of contrast sequences has a more important applied research value in medical clinical diagnosis.

Medical images are usually acquired after the completion of a medical imaging examination, and the process of reprocessing such images is often referred to as post-processing of medical images. At present, almost all imaging devices can directly obtain digital medical images, which provides great convenience for postprocessing work. The application of medical image post-processing is mainly for clinicians or imaging technologists, who usually first apply medical image post-processing software to process medical images and then provide clinicians with more advanced diagnostic information. Medical image postprocessing mainly includes medical image enhancement, segmentation, alignment and fusion, visualization techniques, and data compression [5]. Medical image enhancement is mainly to improve the image contrast, make the image clearer, and improve the visual effect of the image. Image alignment and fusion is the correspondence of multiple images in terms of spatial location to combine information from multiple modalities or multiple periods to provide more diagnostic information, such as aligning structural imaging and functional images in MRI [6]. Data compression is used to reduce the amount of data for storage and transmission. Segmentation and visualization are important elements in medical image post-processing, which play a crucial role in modern medical diagnosis and are directly related to the doctor's diagnostic effect [7]. Usually, doctors are interested in an organ or structure, but medical images also contain surrounding tissues, which makes it difficult for doctors to observe the organ of interest directly. For this reason, image segmentation techniques are needed to separate the organ or tissue of interest from the surrounding tissues, which can facilitate observation on the one hand, and allow measurement and quantitative calculation of organ or tissue information such as volume and organ modeling on the other. Medical image visualization technology, on the other hand, is a better way to display the organ or structure of interest in multiple angles and forms, providing doctors with intuitive diagnostic information and thus improving their diagnostic efficiency and accuracy. Medical image segmentation is often considered as the basis of visualization.

Medical image segmentation and visualization techniques are currently widely studied and applied [8]. Cardiac CT angiography (CTA) technology and MRI are widely used in the diagnosis and treatment of cardiac diseases and neurological diseases of the brain [9, 10], respectively, and rely heavily on segmentation and visualization techniques in their diagnosis [11]. In the case of the heart, for example, techniques such as cardiac segmentation, coronary artery segmentation, cardiac body mapping, and coronary surface reconstruction are usually required. The coronary centerline also has an irreplaceable role in the visualization and reconstruction of the coronary arteries. The techniques of decortication and perivascular gap segmentation are mainly studied on brain MRI images and the segmentation of coronary artery lumen and its visualization on cardiac CTA images. Among them, decriminalization is the basic processing step for brain image segmentation, quantification, and other operations, and decriminalization techniques are used in most structural MRI image analyses, while the perivascular gap is associated with a variety of neurological disorders, such as cognitive impairment, brain developmental diseases, and atherosclerosis. Studying the segmentation of the perivascular gap is a prerequisite for quantitative analysis. Currently, several techniques for visual reconstruction based on CTA data have been used in clinical practice for the diagnosis of coronary artery disease, which includes surface reconstruction techniques (CPR), maximum signal projection (MIP), volume mapping techniques (Volume Rendering Techniques), and multiplanar reconstruction techniques (MPR), especially in the reconstruction of CPR and MPR images. The central line of the coronary artery plays a great role in the reconstruction of CPR and MPR images [7]. Also, the central line of coronary arteries can provide preoperative path planning and intraoperative path guidance for coronary surgical treatments, such as Percutaneous Coronary Intervention (PCI) and Coronary Artery Bypass Grafting (CABG). Therefore, obtaining an accurate coronary centerline is of great importance for clinical treatment. In addition, the central line can also be used as a starting point for the segmentation of coronary arteries.

## 2. Current Status of Research

Since the imaging view of CT completely covers the heart side, the structures presented in the image include a variety of tissues such as bones, muscles, organs, and blood vessels; coupled with the fact that the dose of contrast agent required for imaging affects the picture quality, it makes it further difficult to extract the centerline of the coronary arteries [12]. The existing methods of centerline extraction are divided into three categories according to the degree of human intervention: fully automatic extraction, semi-automatic extraction, and manual extraction [13]. Among these three methods, the manual extraction of the centerline is undoubtedly a simple and reliable method, but when a large amount of data is encountered, the manual extraction method will consume a lot of human and material resources, so it is especially important to study the fully automatic and semi-automatic extraction algorithms [14]. The fully automatic method generally refers to the process of extracting the centerline without any human intervention, and the algorithm automatically extracts the centerline of the coronary artery based on the input data information; the more classical methods include the method proposed by Freiman to further extract the centerline based on the extraction of the coronary vascular tree by fitting the cylindrical model; the semi-automatic method refers to the process of vessel extraction [15]. The semi-automatic method refers to the method in which one or several seed points need to be artificially specified as reference points for centerline extraction, and the algorithm extracts the centerline in the image data based on the artificially provided reference points, such as the method proposed by Kojima et al. to extract the centerline of coronary arteries after segmenting the aorta and coronary arteries and performing 3D reconstruction by using the local gray values of the vessels and the orientation of the vessels to select the starting point of the iteration [16]. The various automatic or semi-automatic methods for extracting the centerline can be classified into the following six types according to the extraction ideas they use: topology refinement-based methods, distance transformation-based methods, tracing-based methods, fast marching algorithm-based methods, deep learning-based methods, and other methods [17]. As an important tool for diagnosing cardiovascular diseases, coronary angiography has an irreplaceable position in clinical practice, so the processing technology for coronary angiography images is always a hot spot for research [18]. Traditional coronary angiography segmentation algorithms can be classified into three types based on the similarity of neighborhoods: boundary-based, region-based, and integrated with specific theories [19]. With the development of the artificial intelligence field and the increase of data volume, the breakthrough of convolutional neural networks (CNNs) in the field of image processing is also bringing great changes to the direction of medical image processing [20]. The main method of convolutional neural networks applied to medical image processing is semantic segmentation, which is the pixel-level classification of images by different model classifiers. In the following section, we present representative methods from traditional and deep learning approaches, as well as the problems in research.

With the development in the field of computer vision, convolutional neural networks have brought revolutionary disruptions to large-scale image processing, and related methods have made great progress in the field of medical image processing. The segmentation of medical images belongs to the category of semantic segmentation in deep learning, which essentially classifies each pixel [21]. In recent years, semantic segmentation has made great progress, and Shi et al. proposed the U-Net network, which has a more regular network structure, and compared with FCN, the more significant change is in the upsampling stage; the upsampling layer of U-Net network also includes many layers of features, and then the features obtained from each upsampling layer are added to the decoder to obtain more accurate features [22]. The U-Net network has been widely used in medical image segmentation, such as cell segmentation, retina, and other blood vessel segmentation fields, and has achieved good segmentation results [23]. The second type is the inflated convolution structure, represented by the Deep Lab network and its two improved versions, and the Refine Net network. Until 2016, Tahoces et al. and two enhanced versions were developed. This network employs convolution with voids rather than traditional convolutional computing, employs various scales to improve spatial resolution of segmentation findings [24], and uses conditional random fields as postprocessing to refine the results [25]. Advances in modern medical imaging technology provide higher resolution medical image data for the diagnostic process while analyzing raw data is inefficient. Visualization technology plays an important role in providing doctors with fast and accurate medical images in a noninvasive manner, providing aids to diagnosis, surgical navigation, treatment guidance, and medical teaching. Curvilinear reconstruction, a technique that uses centerlines to visualize tubular structures, has become a must-have feature of medical workstations, with features such as length retention, allowing the entire vessel or even the entire vascular tree to be displayed on a single image [26]. The main ones currently used are projection CPR, extension CPR, and straightening CPR. Traditional single-vessel CPR plays an important role in vascular diagnosis, while multipath CPR can also play a navigational role. In addition, spherical CPR demonstrates multiple vessels while preserving the spatial structure of the vessels well [27]. The application of virtual endoscopy with face-drawing or body-drawing, on the other hand, is a technique that incorporates a variety of techniques implemented in image processing and virtual reality technology to simulate traditional optical endoscopy, overcoming traditional invasive examination methods, and is mainly applied to organs with cavernous structures, such as the trachea, esophagus, colon, andblood vessels, etc. This technique can provide physicians with navigation within tubular structures with a high degree of realism.

Coronary artery structure is complex, individual vascular variation is large, and its grayscale is affected by abnormal tissues such as plaque, stenosis, and stent, and the grayscale range is large, and coronary lumen segmentation is a difficult task. In this study, the coarse segmentation results of coronary arteries and the vascular centerline calculated from this result have been obtained, and this paper mainly uses these data for further segmentation to obtain the accurate segmentation results of the vascular lumen. The main method is to segment the vessel lumen on the vessel cross section, so the cross-sectional image needs to be acquired first. Based on the straightening reconstruction algorithm, this paper first constructs the straightened image of the vessel and then segments the vessel lumen layer by layer on the cross section. The traditional CPR method, including extension CPR and straightening CPR, is implemented, and then a spherical CPR method is implemented and improved. Firstly, the conventional extended CPR requires projection of the original centerline at a specified angle, and then the original centerline is sampled at equal intervals using the projected trajectory as the standard, followed by determining the extent of the resulting image and filling it with gray values. Straightening CPR requires sampling the original centerline at equal intervals, establishing a local coordinate system along the centerline, and ensuring that the axes are “parallel” to each other, and using a suitable interpolation algorithm to ensure image quality and efficiency. The spherical CPR can display the whole coronary tree on a single image, and the key issues of the algorithm are the acquisition of the centerline envelope surface and the transformation from globe mode to map mode.

## 3. Design of Detection and Extraction of the 3D Arterial Centerline in Spiral CT Coronary Angiography

### 3.1. Spiral CT Coronary Angiogram Preprocessing

Generally, there are two methods for coronary artery centerline extraction: the first one is to directly extract the coronary artery seen in the original image. This has the advantage of not having to segment the coronary artery region. But, the original CT laminar image is affected by noise and there are more irrelevant regions, which often interferes with the extraction results. The other method is to segment the coronary artery first and then use the completed segmented image for centerline extraction. Although this method increases the segmentation step, it has a greater improvement in time and accuracy because there are fewer operations on voxels during centerline extraction [28]. The two proposed algorithms perform centerline extraction in the segmented coronary artery region, so the image needs to be segmented first. Since the imaging principle of CT is X-ray imaging, according to this imaging principle, there is often more noise on the image; in addition, the quality of CTA is influenced by the contrast agent, and there may be blurring in the vascular region, which will often lead to large errors in the segmentation results. So, the necessary denoising and enhancement of the vascular region must be performed before segmentation.

The Anisotropic Diffusion Filter (ADF) is a null domain filter proposed by Gerig et al. Unlike other filters that have only a single filtering effect on the whole image, the anisotropic diffusion filter has different filtering effects in each direction of the image, and these different filtering effects are determined by the diffusion function [29]. The basic theoretical derivation of anisotropic diffusion filtering is presented below, and the process of filtering an image using an anisotropic diffusion filter is

(1) $$\begin{array}{c} u_{t}=u_{xx}^{2}. \end{array}$$

According to the anisotropic diffusion theory, equation (2) can be rewritten as

(2) $$\begin{array}{c} \frac{\partial }{\partial t}u\left(x,t\right)=\mathrm{div}\left(c\left(x,t\right)\Delta u\left(x,t\right)\right), \end{array}$$

where *u*(*x*, *t*) denotes the grayscale of the image, Δ*u*(*x*, *t*) denotes the gradient image of *u*(*x*, *t*), div denotes the scattering operator, and *c*(*x*, *t*) denotes the diffusion function. For the choice of the diffusion function, Gerig and Kubler give two different functions for reference:

(3) $$\begin{array}{c} c_{1}\left(x,t\right)=exp\left(-\left(\frac{\left|\Delta u{\left(x,t\right)}^{2}\right|}{k^{2}}\right)\right), \end{array}$$

(4) $$\begin{array}{c} c_{1}\left(x,t\right)=\frac{\left(\left|\Delta u{\left(x,t\right)}^{2}\right|/k^{2}\right)+1}{1-\left(\left|\Delta u{\left(x,t\right)}^{2}\right|/k^{2}\right)}, \end{array}$$

where *k* is a constant associated with the noise level and the boundary intensity, and here *k*=min|∇*u*| is chosen. Solving the partial differential equation of equation (4) with the 4-neighborhood image as an example, the numerical expression required in the iterative process of the algorithm can be obtained:

(5) $$\begin{array}{c} u\left(t-\Delta t\right)\approx u\left(t\right)-\Delta t\frac{\partial }{\partial t}u\left(t\right), \end{array}$$

where *ϕ* denotes the diffusion flux, and its expression is

(6) $$\begin{array}{c} \phi =c\Delta u. \end{array}$$

In 3D images in the medical field, the tissue structure of the human body can be roughly divided into disk-like, tubular, and patchy structures. Therefore, the Hessian matrix of a pixel can be calculated to determine the shape of the tissue structure to which the pixel belongs based on the magnitude, and positive and negative cases of the absolute value of its eigenvalue. *N* means almost zero, *L* means small absolute value, *H* means large absolute value, and “+/−” indicates the positive and negative cases of the eigenvalues, which are indicated by the brightness of the blood vessels: bright blood vessels are negative and darker ones are positive. Therefore, it can be seen from the Figure 1 that the absolute value of *λ*1 should be small and close to 0; the absolute values of *λ*2 and *λ*3 should be much larger than *λ*1, and the positivity and negativity are the same, so the relationship of the eigenvalues of the vascular structure is expressed by mathematical expressions, as shown in Figure 1.

Due to the small amount of coronary angiography image data, data enhancement of sample images is needed to enhance the image quality to improve the generalization ability of the neural network model. In this article, firstly, specular symmetry, image rotation, and contrast stretching methods are used to enhance the quality of the sample images. Subsequently, the full convolutional segmentation network VGG-seg is proposed, which is based on a modification of the VGG-16 network by removing the final fully connected layer and deconvoluting after each pooling layer, and linearly summing the results of the deconvolution of each output layer separately to classify each pixel. In the learning process, the pretraining results on ImageNet were first used as the starting network, and then this initialized model was applied to the fully convolutional segmentation network, and 109 X-ray angiography sequences from the training set were used for training to extract blood vessels; finally, the model was tested using 40 coronary angiography sequences from the test set to achieve real-time vessel segmentation [30]. In deep learning, the number of samples is generally in great demand, and the more the number of samples and the richer the variability, the stronger the generalization ability of the model and the better the effect of the network model obtained by training. Fully convolutional neural network-based coronary angiography image vessel segmentation requires a large amount of real patient data to train the network, and it is very difficult to obtain sufficient sample sets, so image enhancement of existing data is required to lay a good foundation for the subsequent model training.

To increase the difference in gray level between pixels and highlight the blood vessels, enhancement of the image is achieved by using the gray-level change method. The grayscale transformation method alters the contrast of an image by changing the range of grayscale levels and is a histogram change-based method. In theory, the value range of image grayscale is [0, 255], that is, a total of 256 levels, and in the imaging process, due to some factors, such as lighting and equipment quality, the grayscale level of the image is often less than 256, that is, the grayscale range of the image will be compressed to [0, 255] within a certain subinterval, which is the fundamental reason for the low contrast of the image. To increase the contrast, we need to increase the grayscale value range, that is, to map the smaller grayscale range to a larger range by the value range stretching operation. The general case of the grayscale mapping function is defined in equation (7).

(7) $$\begin{array}{c} f=\frac{d+c}{b-a}\left(g+a\right)-c. \end{array}$$

Based on the results of the above preprocessing, the study of the coronary angiography sequence segmentation method will be started in the following. Image segmentation is a prerequisite for image recognition and analysis, to divide the image into multiple parts according to the needs and make it easy to analyze. The essence of image segmentation is to cluster the pixels containing the same characteristics into one class based on their characteristics. A convolutional neural network automatically extracts features by simulating the process of human brain cognition for the ultimate purpose of classification or prediction [31]. The development of convolutional neural networks has revolutionized the field of image segmentation by automatically extracting features of images through multilayer convolutional computation to achieve the pixel-level classification of images, i.e., to achieve image segmentation. Convolutional neural networks have automatic, fast, and accurate characteristics in processing large-scale image data, and have unparalleled advantages over traditional methods, and have achieved wide application in the field of image segmentation.

The human head is protected by the cranium so that its morphological structure is not as susceptible to deformation as the heart and remains largely stable, and therefore can be considered for cranial debridement using an alignment method. Many alignment-based decriminalization methods exist, which are often computationally intensive but have stable results. In this section, the initial mask of the brain parenchyma is first calculated using the alignment method, and then the initial mask is improved using the level set method to generate the final mask.

Image alignment is the process of locating a spatial transformation that maps points in one image to points in another image, connecting points in both images that correspond to the same spatial position, and aligning the two images in a specified space. For medical images, the result of alignment should make the points with diagnostic significance in both images match. Taking the two-dimensional image alignment as an example, as shown in Figure 2, the alignment process can be described as equation (8) by noting the reference image and the image to be aligned as *I*_*r*_ (*x*, *y*) and *I*_*x*_ (*x*, *y*), respectively.

(8) $$\begin{array}{c} I_{x}\left(x,y\right)=g\left(I_{r}\left(T\left(x,y\right)\right)\right), \end{array}$$

where *T*(*x*, *y*) denotes the spatial transformation and the function *g*(*I*_*r*_(*T*(*x*, *y*))) denotes the grayscale transformation; usually, the grayscale transformation is not necessary and the key is to find the spatial transformation between the two images. The solution of the spatial transformation is usually treated as an optimization problem, which is usually achieved by iteration.

The image alignment process generally consists of two steps: first, extracting the feature information of the image to form a feature space; then, defining a similarity criterion from the feature space and determining a spatial transformation so that the image can achieve the defined similarity after the transformation. The computation of the spatial transformation is generally done using optimization methods, and the process of generating the alignment image often requires image grayscale interpolation. Therefore, feature space, similarity measure, spatial transformation, optimization method, and interpolation method are the five major elements of image alignment. The feature space can be generally divided into three categories, including feature points, feature curves or feature surfaces, and pixel values. The commonly used similarity measures include meaning square error, correlation, and mutual information. The definition of alignment is based on spatial geometric transformations, which can be divided into rigid and nonrigid transformations according to the different ways of image deformation. Rigid transformations include translation and rotation, which are commonly used in the alignment of human brain images; nonrigid transformations include scaling, affine transformation, projection transformation, and curve transformation. The alignment process is usually transformed into a polar solution problem, using an optimization search algorithm such as the gradient descent method. Commonly used grayscale interpolation methods are linear interpolation, nearest-neighbor interpolation, and spline interpolation. To achieve better computational efficiency and alignment quality, different alignment methods should be selected according to the image deformation mode.

The coronary artery system is composed of three layers of vascular membrane structures, the inner, middle, and outer membranes, in order from the luminal surface (innermost layer) outward, which make up the coronary artery, an elastic, contractable, and expandable system of tubes. The cross section perpendicular to the direction of blood flow in this system can always be considered as a subcircle. Depending on the direction of growth of the coronary arteries, the entire vascular tree can be considered as the root system of the plant. The coronary arteries originate from the root of the ascending aorta, so the ascending aorta can be compared to the main root in the root system. The left and right coronary arteries and the many vessels emanating from them, such as the left circumflex branch, the obtuse marginal branch, the diagonal branch, and the left anterior descending branch, can be compared to the lateral roots in the root system. In the coronary artery system, vessels are usually three-branched or even four-branched, but those with diagnostic value in clinical practice are usually vessels larger than 1.5 mm in diameter, which are often two-branched vessels.

### 3.2. Contrast Map Centerline Extraction

The extraction of the coronary artery centerline can start from a specified position, and according to the predefined conditions, it is assumed that a small elastic ball is rolled in the direction of blood flow in the coronary artery, and the position of the ball center and the radius size are adjusted in real-time according to the current position until the predefined conditions are met or the largest internal contact ball at that position is found to complete the search at the current position. Then, the ball continues to roll in the direction of blood flow and searches the whole vessel one by one according to the above method until the search is completed. When the sphere encounters a bifurcation point of a coronary artery, the sphere may split into two spheres and then complete the search of the vessel tree in parallel with the above steps [32]. During this process, the positions of the centers of all the maximal internal spheres are recorded, and a curve is formed, which is the centerline of the vessel. However, it has been a difficult problem to determine the location of the center of the next internal sphere when searching for the centerline using the maximum internal sphere. One idea to solve this problem is that a point on the sphere of the previous sphere can be selected as the center of the next inner-junction sphere according to the course of the vessel, and the inner-junction sphere at this point must be larger than the inner-junction sphere generated by other voxels on the sphere and cannot be contained by the intersection of other inner-junction spheres. The model of the maximum inner-junction sphere in the vessel is shown in Figure 3.

An object is usually considered to be sampled uniformly in 3D space, where a voxel is the smallest unit, and a voxel contains an Object voxel and a Background voxel. In this method, the target voxel is considered to have 26 neighbors and the background voxel is considered to have only 6 neighbors. In addition, there is a class of Boundary voxels among the target voxels, which are the target voxels with 6 adjacent background voxels, and these boundary voxels form the boundary of the object. For an arbitrary voxel *p*, it can be defined that its 26 neighbors in space can be split into F-neighbors, Edge-neighbors, and V-neighbors, which are shown in Figure 4. The figure shows that there are 6 F-neighbors of any voxel *p* (centrally located voxel), which share their 6 surfaces with *p*; 12 E-neighbors of *p*, which share their 12 ribs with *p*; 12 E-neighbors of *p*, which share their 12 ribs with *p*; and 12 E-neighbors of *p*, which share their12 ribs with *p*. Some voxels share their 8 top angles with *p*, which make up the V-adjacent voxels of *p*.

The distance transform can be used to calculate the distance between a pixel point in an image and an area block by using a neighborhood mask, and then the global distance of the image is approximated using the local distance on the way to propagation. To efficiently process 3D data, the target is represented as an octree structure and no background voxels in the image are stored. Since it is not efficient to traverse the octree in array order, the algorithm uses a technique of propagating the distance transform continuously inward from the boundary voxels to increase the efficiency of the traversal, which requires two assignments of the distance transform to the target voxels.

(9) $$\begin{array}{c} L\left(W\right)=\sum_{i}\beta y_{j}\ln\;P\left(y_{j}=11X\right),\\ \sum_{i}\beta y_{j}\ln\;P\left(y_{j}=11X\right)=1-\beta \sum_{i}\beta y_{j}\ln\;P\left(y_{j}=11X\right), \end{array}$$

The main purpose of the first assignment is to find the boundary voxels in the target region. The 26 adjacent voxels of each target voxel are checked for the presence of background voxels, and if they exist, their distance transform values are assigned according to the following rules and the voxel is classified as a boundary voxel.

In the initialization phase of the algorithm, a list is created for the distance transformation values of each voxel belonging to the target region according to the setup requirements of the algorithm; this list is used to store a pointer to find a node in the octree, and each node in the octree represents the distance transformation value of each voxel, which is found by the values in the list. In the first pass, the circular queue initializes the list with the distance transform values 3, 4, and 5, and the queue starts with 3, assigning the corresponding distance transform value to each voxel belonging to the target region. Starting from the second pass, the boundaries will be shrunk inward as shown in Figure 5.

The essential voxels that make up the skeleton lines of the target region can be determined by calculation so that these voxels can be identified using the property that the skeleton lines can reconstruct the original shape. This means that it is possible to reconstruct the approximate shape of the original figure based on the voxels on the skeleton line and their distance transformation values, but it is not enough to have only a rough skeleton line if the precise shape is to be reconstructed; the skeleton line must also contain all the shape features of the original figure [33]. Therefore, it is more important to preserve the skeleton line accurately in the region where the shape changes or the curvature changes suddenly, and the more accurate the skeleton line is, the more accurate the reconstruction can be.

(10) $$\begin{array}{c} \beta =\frac{Y^{2}}{X}. \end{array}$$

During this traversal, when the program runs to a certain instant, the point being processed with a distance transformation value of *k*(*k*=3,4,5) can only have a distance transformation value of *k*+3, *k*+4 or *k*+5 for its neighboring voxels. Iterate through the list at the beginning of the queue and estimate the distance transformation value for all the target voxels adjacent to the boundary voxel. At this point, the distance transformation value is the sum of the list value and the local distance increment, and the size of the increment is 3, 4, or 5 depending on the type of the adjacency. If the new distance transformation value is lower than the value in the current list, the voxel is added to the list corresponding to the new value, and the voxel becomes the new boundary voxel, and the original boundary voxel becomes the background voxel. After processing the list of neighboring voxels of the current boundary voxel, the same judgment process is performed for the neighboring voxels of the next boundary voxel until all the boundary voxels of the layer are traversed and the calculation stops, i.e., no more distance transformations of the neighboring voxels of the boundary voxels need to be assigned, as shown in Figure 6.

To find the nonwitness voxels that can complete the graph reconstruction, it is necessary to filter the 26 adjacent voxels of all target voxels. Since all nonwitness voxels have maximal inner-joining spheres, no single maximal inner-joining sphere of a neighboring voxel can completely contain the sphere of nonwitness voxel *p*. However, according to the above, the maximal inner-joining sphere of a nonwitnessing voxel can be contained in the concatenation of the maximal inner-joining spheres of several other voxels. If such voxels exist, their maximal inner-joining spheres must be at least as large as the inner-joining spheres of *p*, which means that the value of their distance transformation should be greater than or equal to *DTp*. There is another simpler way to filter for neighboring voxels. The significance of this is that if several of the neighboring voxels of *p* have higher values of the distance transformations, the inner-joining spheres of *p* may be contained in the merged set of inner-joining spheres of those voxels.

The core idea of the deep convolutional neural network is to learn about a large amount of data and capture their features by building a model containing three or more hidden layers, to reach the purpose of classification or prediction for new input data. In a deep convolutional neural network, the original image as a whole or its local part is used as the input of the bottom layer, and the information of the original image is passed to different layers at the back through convolutional operations of certain size templates, and each layer extracts the significant features in the image through convolutional operations of different sizes, and finally calculates the classification probability of pixels with certain features through activation functions to achieve classification. According to the above process, CNN mainly contains the input layer, convolutional layer, pooling layer, fully connected layer, activation function, and output structure, as shown in Figure 7.

The input layer is the input to the whole convolutional neural network, which generally represents the pixel matrix of a picture in a convolutional neural network that processes images. As shown in Figure 8, the uppermost part represents a picture (RGB 3D). The length and width of the 3D matrix represent the size of the image, while the depth of the 3D matrix represents the color channel of the image. For example, handwritten characters are recognized as black and white images with a depth of 1. In the RGB color model, the depth of the image is 3. Starting from the input layer, the convolutional neural network transforms the matrix of the previous layer into the matrix of the next layer through different neural network structures until the final fully connected layer.

The pooling layer is a computation that compresses the individual submatrices of the input tensor. It is like the computation of convolution, which is also performed on an image utilizing templates of a specific size, but the difference is that the final output of each template has only one value, which is usually the maximum value in the image within the range of the template (at this point called maximum pooling) or the average value (at this point called average pooling). The effect of the pooling layer is to combine similar features within a certain range, which can be very effective in reducing the size of the parameter matrix and thus the number of parameters in the final fully concatenated layer, thus speeding up the computation and having the effect of preventing overfitting.

The power of deep convolutional neural networks lies in their ability to automatically extract features through a combination of multiple convolutions and pooling while being able to learn features at multiple levels. Among them, the front convolutional layer has a small range of receptive fields and can learn features of local regions of the image, while the back convolutional layer has a larger range of receptive fields and can learn more abstract features, which are less sensitive to the position and size of objects. These abstract features are helpful for classification but become difficult for giving object contours and accurately segmenting objects due to the loss of details. When traditional convolutional neural networks perform segmentation, to predict the class of a pixel, they need to be trained and predicted using blocks of images within a certain range of its neighborhood, which requires large storage and is inefficient in terms of computation [34]. To solve this problem, Jonathan Long et al. proposed Fully Convolutional Networks (FCN) for image segmentation. The idea of FCN is to use up-sampling of abstract features to predict the class of each pixel of the original image, which is a way to convert the macroscopic (image-level) segmentation problem into a microscopic (pixel-level) classification problem.

FCN is a classification of pixel-level labels, and the segmentation problem of the whole graph is achieved by the classification of all pixels. Unlike CNN, which uses fully connected layers at the end to obtain fixed-length feature vectors for prediction one by one, FCN removes the last fully connected layer and performs deconvolution calculation on the output of the last convolution layer to obtain a feature map of the same size as the original map, which also restores the spatial characteristics of the original map, where each pixel in the generated feature map may be used as a sample for training to predict the class of each prediction of the category of each pixel, and so the entire graph can be segmented. The network finally removed the fully connected layer and recovered the image size using deconvolution to predict each pixel category, which resulted in the semantic segmentation of the image.

## 4. Analysis of Results

### 4.1. Experimental Results

The topology refinement algorithm described in this chapter is used to extract the centerline of the vessel after 3D reconstruction and to compare the effect of performing the fine branch removal operation on the extraction accuracy.  Figure 9 shows the results of centerline extraction using the algorithm in this section in a single vessel, where a right coronary artery is selected in Figures 9(a) and 9(b), and a left anterior descending branch is selected in Figures 9(c) and 9(d). Figures 9(a) and 9(c) show the results of centerline extraction without fine branch removal; Figures 9(b) and 9(d) show the results of extraction with fine branch removal. The gray part of the figure shows the reconstructed coronary artery region, and the blue curve in the middle is the extracted central line. By comparing the four figures, it is easy to find that the Dijkstra algorithm-based fine branch removal method used in this chapter has a good limiting effect on the fine branches generated in the extraction process, greatly reducing the burrs on the centerline, making the extracted centerline smoother and more consistent with the actual shape of the centerline.

To demonstrate that the Dijkstra-based minutiae deletion algorithm can effectively improve the accuracy of the topology refinement algorithm in a single vessel, all vessel data in the dataset were extracted from the centerline separately according to the evaluation criteria proposed in Section 3.2, and then the extraction results were quantified and analyzed, and the results of six vessels were randomly selected for display.  Figure 10 shows the results of centerline extraction without fine branch removal, the results of fine branch removal for the extracted skeletal lines after completing the topological refinement in twelve directions. The six vessels include a right coronary artery (RCA3), two left anterior descending branches (LAD1, LAD2), a left gyral branch (LCX2), a sharp-edge branch (MA1), and a posterior descending branch (PDA2).

Also, in this section, CTA data were used to test the effectiveness of the algorithm for centerline extraction in coronary vascular trees. The number of images used varies between 250 and 350 for each case with a single image size of 512 × 512, a spatial resolution of 0.38 mm, a layer thickness of 0.5 mm, and a minimum reconstructable thickness of 0.6 mm; the bulb voltage used for scanning is 100 VK, and the convolution kernel for 3D reconstruction is Bv36d. The results of the complete coronary vascular tree centerline extraction are shown in Figure 11. The results without fine branch elimination are shown, and the results after fine branch elimination are shown. The gray part of the figure shows the reconstructed vascular region, and the thicker part above is the ascending aorta, from the end of which the coronary arteries diverge into two branches, left and right. Because the centerline of the ascending aorta is not within the scope of this study, its centerline was not extracted. After comparing the two figures, it can be found that the algorithm has a better extraction of the centerline of the coronary vascular tree, and a more complete centerline is also preserved for the end bifurcation part of the left anterior descending branch; after the fine branch elimination, the burr part in the right coronary artery in the figure is effectively restricted, which makes the centerline of the complete vascular tree smoother and more consistent with the actual situation of the centerline. At the same time, this experiment also proves that the algorithm in this chapter has strong robustness and can complete the extraction of centerlines of multiple heeled vessels simultaneously.

Usually, medical images should keep the size and shape of the original structure as much as possible. So, the projection curve is sampled at equal intervals in the process of straightening the collinear, with each sampling point corresponding to one line of the output image. The output image is then sampled in grayscale, usually using trilinear interpolation for grayscale sampling. In extended CPR, the sampled surface defined by the centerline and the direction of interest is essentially a column surface, the line in the direction of interest is the mother line of the column surface, and the curve obtained by projecting the centerline along the direction of interest is the collinear line of the column surface. The collinear dimension of the surface is flattened and then sampled in grayscale from the original body data space to obtain the extended CPR image. As shown in Figure 11, the green arrow is the direction of interest, which is also the centerline projection direction of the extended CPR; the red curve is the vessel or its centerline; and the dashed line on the right side of the plane perpendicular to the green arrow is the projection of the centerline on the plane, which is the collinear line of the column surface; and the final CPR image is obtained by straightening the projection curve.

### 4.2. Algorithm Results

The main goal of the model training process is to achieve the distinction between foreground and background, i.e., vascular, and nonvascular. One hundred and nine coronary angiography sequences were randomly selected as the training set to train the segmentation model. Each sequence contains 30–50 frames, and the size of each frame is 512*∗*512. Stochastic gradient descent (SGD) is used as the optimization function for the iterations, i.e., only one sample is randomly selected from the total data at a time to update the iteration function with a momentum of 0.9. The initial learning rate is set to 0.001, and then gradually decreases. After training, the generated model is saved as a segmentation model, which enables the segmentation of foreground (vascular) and background (nonvascular). In the training, we found that there is a balance between the time required for prediction and the number of model iterations. Within a certain range, as the number of iterations increases, the segmentation effect is better, while the waiting time is longer. For the balance consideration, the segmentation result of 400 iterations' output is chosen in this paper. The following figure shows the performance curve of the network training process, where loss is the loss function; Dice is the parameter to judge the segmentation effect of the network, the closer to 1 the better the segmentation effect, which will be explained in detail in Chapter 4, as shown in Figure 12.

In the training process, two methods, data enhancement and adding dropout layers, were utilized to prevent overfitting. For data augmentation, we perform random mirror symmetry on the coronary angiography experimental data with 50% probability, followed by random rotation with 50% probability, and finally, the brightness change with 50% probability, and all the data obtained from the augmentation process are input to the network for training. For the dropout layer, the intuitive explanation is to deactivate some nodes in the network randomly, and after several different dropouts, it is equivalent to training several different networks, which is the embodiment of the idea of integrated learning model and realizes the fusion of models in the same network with lower space occupation than the fusion of multiple networks. The random deactivation probability used in this paper is 0.5, and this value is found to minimize the convergence of the loss function in the experiments. Finally, data from 40 patients are used as test set data in this paper to test the performance of the model.

Figure 13 shows the comparison of the results of the two centerline extraction algorithms proposed in this paper with the abovementioned twenty-six directional refinement algorithms. The comparison results used in the table are obtained by taking the average of all the experimental results of the three algorithms after experimenting with all the labeled vessel data. Analyzing the data in the table, we can see that the TDTT algorithm proposed in this paper has improved the overlap rate by 5.4% compared with the MIBTT algorithm; the TDTT algorithm has reduced the average distance to the actual length by about 0.16 mm; the TDTT algorithm has improved the overlap rate before the first error by 63.3% compared with the MIBTT algorithm; the running time of the TDTT algorithm is about 9% of that of the MIBTT algorithm. The average running time of the MIBTT algorithm is 5.217 seconds, which can meet the design requirements of CAD systems in clinical practice.

Comparing the results of centerline extraction based on the twenty-six directional topology refinement algorithm with the TDTT algorithm, we get to see that the overlap rate of the TDTT algorithm is 49.7% higher than that of the algorithm; the average distance is only 20% of that of the algorithm; the overlap rate before the first error is 3.24 times of that of the algorithm; and the extraction time is only 5% of that of the algorithm. After analysis, it is found that the defect of the topology refinement algorithm based on the twenty-six directions is that it does not eliminate the fine branches of the extracted centerline, resulting in a large number of burrs on the extracted centerline, which are composed of several or even dozens of voxels, and due to their existence, the overlap rate of the extracted centerline is greatly reduced, and the average distance between the extracted and labeled points appears to increase dramatically. This indicates that the algorithm in this chapter is more suitable than this method for coronary centerline extraction in terms of both running accuracy and running time. By comparing the results of the MIBTT algorithm and the twenty-six direction-based topology refinement algorithm, it is easy to find that the performance of the MIBTT algorithm also has a substantial lead. So, the two coronary centerline extraction algorithms proposed in this paper are more suitable for coronary centerline extraction than the twenty-six direction-based topology refinement algorithm. As the more classical coronary centerline extraction algorithms, the overlap rates of the proposed algorithms are 0.847 and 0.670, respectively, and compared with this result, the two algorithms proposed in this paper have higher extraction accuracy in coronary centerline extraction.

A method of coronary artery centerline extraction based on a twelve-directional topology refinement algorithm (TDTT) is proposed. The algorithm performs a refinement operation on the reconstructed coronary artery region based on the segmentation of the original image to extract the centerline while maintaining the original topology of the coronary artery as much as possible. At the end of the refinement algorithm, Dijkstra's algorithm is introduced to trim the fine branches in response to the phenomenon of burrs on the centerline during the extraction process, so that it can reflect the actual shape of the coronary artery centerline more realistically. This chapter also evaluates the centerline extraction results of a single vessel in terms of overlap rate, average distance, overlap rate before the first error in the vessel, and running time, and shows the algorithm's extraction results for the centerline of a complete vessel tree. Finally, the two algorithms proposed in this paper are compared, and the results show that the algorithm in this chapter has certain advantages; meanwhile, the algorithm proposed in this chapter is compared with the classical topology refinement algorithm based on twenty-six directions, and it is proved that the algorithm in this chapter is more suitable than this method for extracting the centerlines of coronary arteries.

## 5. Conclusion

For coronary artery centerline extraction, the basic idea of the study is generally to first segment the original CTA to obtain the coronary artery region, then perform 3D reconstruction, and finally extract the coronary artery centerline in 3D space. The first part of this study follows this idea to segment the CTA. Since the imaging principle of CT is X-ray imaging, the image contains a large amount of scattered noise, and the image is first filtered by an anisotropic diffusion filter, which has the advantage of different smoothing degrees for each direction of the image compared with other filters that only have a single smoothing degree for the image; then, the Frangi vessel enhancement function based on the Hessian matrix is used to filter the image. Enhancement function based on Hessian matrix is then used to enhance the edges of the tubular structure in the image; finally, the coronary artery region in the image is segmented using the region growth method, and the holes generated in the segmentation are filled using the hole filling technique to obtain an accurate segmented image. Based on the completion of segmentation, this paper proposes a method of coronary artery centerline extraction (MIBTT) based on the tubular tissue inner splice ball model. The algorithm first uses two distance transformations to complete the initial contraction of the 3D blood vessels; the first distance transformation is to complete the boundary search of the original figure, and the second traverses the values of the distance transformations of all voxels to contract the original figure to the inside to reduce the computational consumption in the next step of the process; then, the nonwitness voxels are used to construct the maximum internal junction sphere model to find the skeletal voxels that can reflect the shape of the original figure. These initially extracted skeletal voxels are optimized on the skeletal line using a dichotomy-like principle to obtain the final coronary artery centerline. The experimental results show that the algorithm has a good result in extracting the coronary artery centerline, with an overlap rate of 0.934, an average distance of 2.477 pixels from the reference position, an overlap rate of 0.508 before the first error, and an average running time of 5.217 s. However, the algorithm also has shortcomings in that the centerline of the vessel is not well preserved at the two ends of the vessel, and the centerline of the vessel is not well preserved when dealing with a horizontally oriented vessel. However, the algorithm has the disadvantage that the centerline of the vessel is not well preserved at the two ends of the vessel, and it is prone to incomplete extraction when dealing with vessels with horizontal orientation.

## Figures and Tables

**Figure 1:** Ellipsoidal model.

**Figure 2:** Image alignment principle.

**Figure 3:** Model of the inner joint ball.

**Figure 4:** Schematic diagram of the three kinds of adjacencies.

**Figure 5:** Model of the inner jointed ball of voxel *p*.

**Figure 6:** Detection of calcified plaque.

**Figure 7:** Composition structure of the convolutional neural network.

**Figure 8:** Convolution operation in images.

**Figure 9:** Centerline extraction results.

**Figure 10:** Results of coronary artery centerline extraction without removing fine branches.

**Figure 11:** Results of coronary vessel tree centerline extraction.

**Figure 12:** Optimized network after model training.

**Figure 13:** Comparison of algorithm results.

## Data Availability

The labeled dataset used to support the findings of this study is available from the corresponding author upon request.
